# Board characteristics, institutional ownership, and investment efficiency: Evidence from an emerging market

**DOI:** 10.1371/journal.pone.0291309

**Published:** 2024-02-07

**Authors:** Shahid Ali, Muhammad Farooq, Zhou Xiaohong, Martina Hedvicakova, Ghulam Murtaza

**Affiliations:** 1 School of Economics and Management, Anhui Polytechnic University, Wuhu, Anhui, China; 2 Institute of Business Management & Administrative Sciences, The Islamia University of Bahawalpur, Bahawalpur, Punjab, Pakistan; 3 Department of Economics, Faculty of Informatics and Management, University of Hradec Králové, Králové, Czech Republic; 4 Department of Commerce, The Islamia University of Bahawalpur, Bahawalpur, Punjab, Pakistan; Yunnan Technology and Business University, CHINA

## Abstract

This study investigates the impact of board governance mechanism on investment efficiency (IE) in PSX-listed firms. The study also examines the role of institutional ownership (IO) in board-IE relationships. In addition, we extend our analysis to re-examine this relationship by splitting the sample into two groups, i.e., the introductory phase of corporate governance (CG) i.e., 2004 to 2013, and revised codes of CG (2014 to 2018) to examine the impact of these separately on IE. The sample data comprises 155 non-financial PSX-listed firms from 2004 to 2018. IE is measured using firms’ growth opportunities. The random effect model is used to test the study’s hypotheses. A robustness test is also performed to validate the study’s findings. The paired-sample t-test results show a significant improvement in IE after revising the CG codes in 2012. According to the regression results, board size has a significant direct, whereas board diversity has a significant inverse effect on IE. Regarding moderating effect, IO was found to moderate the relationship between board independence and IE significantly. Furthermore, it was discovered that following the issuance of revised CG codes-2012, the level of board independence and diversity increased in PSX-listed firms; however, only diversity positively impacted IE, and board independence had no impact on IE from 2014 to 2018. Despite the issuance of revised CG codes-2012, the level of CG among PSX-listed firms is low, which is a source of concern for regulators such as the Securities and Exchange Commission of Pakistan.

## 1. Introduction

This study investigates the impact of one of the important aspects of corporate governance (hereafter, CG), namely board characteristics, on investment efficiency (hereafter, IE). In addition, we aim to examine the moderating impact of institutional ownership (hereafter, IO) in the board characteristics-IE relationship. Furthermore, in additional analysis, the current study extended the existing CG literature by dividing the sample period into the introductory phase of CG-codes-2002 (period from 2004 to 2013) and revised CG codes-2012 (period from 2014 to 2018) to examine the level of investment efficiency in two periods separately and to examine what role revised CG-codes has on board characteristics-IE relationship. The term "investment efficiency" refers to how well companies invest in their assets. Li and Wang [1] define an organization’s IE as a "project with a positive net present value (NPV)." McNichols and Stubben [2] added that a firm’s investment decision is based on several predefined criteria such as expected return, projected future growth, and projections about product future demand in the market. It is based on judiciously using capital flows, which involve optimal investing that leads to growth, creating more investment opportunities, and enhancing financial capabilities [3]. A firm that invests efficiently is more likely to enjoy superior financial performance since higher IE translates into more efficient use of assets and, ultimately, better firm performance [4]. IE is essential for firms’ long-term growth and country-level economic progress [5].

Moreover, determining capital allocation has been attracting attention continuously in the literature because it concerns fundamental policy toward market development [6]. Therefore, understanding the factors that affect IE will help policymakers to develop policies that improve stakeholders’ confidence in the capital market [7]. Low IE stifles not only corporate growth but also influences overall economic growth. Overinvestment or underinvestment is a phrase used to describe inefficient corporate investment activity. Overinvestment is defined by Biddle, Hilary [8] as a firm’s investment in negative NPV projects, whereas underinvestment is defined as a firm’s failure to invest in any NPV project [1]. Scholars use agency theory to explain this inefficiency in investment. According to the agency theory, managers make investments blindly to pursue personal benefits, such as greater control over resources, without considering the efficiency of the investment [9]. Managers, on the other hand, according to Aggarwal and Samwick [10], will occasionally postpone investing in positive NPV projects if they have private benefits. Managers want to work less, yet investing requires them to spend more time supervising the company’s operations.

The Asian financial crisis (1997–98) affected the majority of Southeast Asian countries, particularly Pakistan. The crises revealed that a lack of accountability and transparency, as well as a poor capital structure, were major contributors to the crisis, implying an increased need for good corporate governance. There is a widespread agreement that effective CG leads to higher investment performance by mitigating the agency problem and information asymmetry between insiders and outsiders [11]. This lack of information makes it more expensive for managers to keep an eye on outsiders [12]. On the other hand, it may cause managers to over-invest when they have extra cash on hand [13], which may not be good for shareholders in the long run [14–16]. By reducing the agency costs associated with overseeing and controlling management, good corporate governance also enhances investment decisions. According to Chen, Hope [17], an effective governance mechanism in an organization leads to higher IE, which in turn increases firm value. Gill, Sharma [18] claim that a good governance mechanism increases firm IE, allowing firms to penetrate local and international markets. Board structure is one of the key components of corporate governance and is measured by factors like the total number of directors, independent members, the percentage of busy directors, board committees, etc. As a CG mechanism, the board structure includes various elements that can ensure effective CG implementation and increase firm value [19, 20]. A competent board of directors is regarded as crucial to the competitiveness and health of a company. Prior studies have demonstrated that the characteristics of the Board of Directors affect the investment efficiency of corporations [4]. According to Kim, Burns [21], the investment decision is one of the most important strategic decisions made by the board of directors. The board of directors is responsible for ensuring that the organization’s finances are managed efficiently and effectively to achieve its goals. Although the finance manager controls investment decisions, the board of directors advises on fund allocation in terms of total assets, firm asset structure, and the consequent risk profile of the options [22]. Watson and Head [23] remarked that the ultimate success and well-being of the company are in the hands of the board of directors. However, the rationale for this relationship remains obscure.

According to Assidi [24], the ownership structure has a significant impact on the structure of the company’s highest authority, mode selection, and the effectiveness of the company’s strategic decision-making process like IE. Institutional investors (IO) have become the largest shareholders in firms operating in developed countries over the last two decades, and their market capitalization in Asia and Latin America is rapidly growing [25]. IO are rapidly defining the new financial landscape and playing a significant role in global capital markets [26]. The presence of IO is a highly active CG control mechanism [27]. Influential institutional ownership can influence the relationship between board characteristics and IE in two ways. On the one hand, by promoting the optimal allocation of business resources and through effective monitoring of managerial activity, powerful institutional investors can significantly strengthen the monitoring mechanism of board governance mechanisms, leading to a higher level of IE. In contrast, institutional owners can subdue IE by inciting conflict between shareholders and non-investing stakeholders. As a result, the presence of IO is predicted to have a major impact on an organization’s board governance system. As a result, the conflicting impact of IO on board governance mechanisms motivates us to expand our primary investigation, i.e. board characteristics-IE, by incorporating the moderating impact of IO between the two.

Because information asymmetry and agency issues are worse in emerging economies than developed countries, they must address corporate investment inefficiencies [6]. According to the World Bank, one of the top five issues confronting more than 26,000 firms in 53 developing countries is the cost and availability of debt and equity financing [28]. The ownership of publicly traded companies in emerging markets is highly concentrated. Family members in most emerging market firms hold key executive and non-executive positions [29]. Most of the shares in most companies listed on the Pakistan Stock Exchange (PSX) are held by family members [30]. Most research on board characteristics and IE has been conducted on firms listed in developed markets (e.g., [3, 31–33]. Board characteristics may influence corporate IE in emerging economies differently than in developed economies due to institutional differences. Finally, following global trends, the majority of developing nations have taken institutional and regulatory steps to strengthen corporate governance mechanisms.

Furthermore, Pakistan’s socioeconomic behavior and institutional framework differ from that of the West and other countries in the region [34]. A controlling or founding family owns most of the shares of PSX (Pakistan Stock Exchange) listed companies [30]. Furthermore, Pakistan’s unstable democratic system has created an unfavorable political and legal environment [35], which fosters corruption and ineffective government (Transparency International). During the last two decades, Pakistan’s government effectiveness and regulatory quality index ratings have also declined, according to the World Bank. As a result of these conditions, the economy engages in immoral and opportunistic behavior [36]. Because of the distinctions mentioned above, the current study represents a unique opportunity to examine the relationship between IO, board characteristics, and IE. The purpose of this paper is to answer the following questions: What is the impact of board characteristics (board size, board independence, board activity, and board gender diversity) on investment efficiency (IE) of PSX listed firms, and how is this relationship moderated by the level of institutional ownership (IO) of respective firms?

Following Biddle [8] and Gomariz and Ballesta [37], we used an IE model based on growth opportunities. Board characteristics include board size, independence, activity, meeting, and diversity. The control variables of the study are firm size, profitability, leverage, and IO. Based on the Houseman test, we used the Random Effect Model (REM) to investigate board characteristics and IE. Based on REM, we found that board size positively impacts the IE of sample firms, while board activity has a negative impact. We also test the moderating effect of IO on board characteristics-IE. IO moderates board independence-IE positively. Further, the findings show that there has been no significant improvement in IE since the issuance of revised codes in 2012, indicating the need to strengthen the governance mechanism in PSX-listed firms in the true spirit.

The article contributes to the emerging literature in multiple ways. First, our paper adds to previous research primarily focused on developed countries [38, 39]. However, due to differences in firm CG and financial structure, as well as differences in countries’ political, social, and legal systems, and differences in ethical attitudes and approaches to investment, the corresponding results for developed countries may not be generalizable to developing economies. As a result, this issue is being researched in developing countries, particularly Pakistan, where the corporate sector is characterized by director interlocking, pyramid ownership, and proxy directorship. Second, we have a single-tier board structure in Pakistan. One-tier board structure governance differs significantly from two-tier board structure governance [40–42]. This model’s institutional settings and litigation environments are thought to affect market investment behavior. The results of this study show how the board of director’s characteristics affects PSX listed firms’ investment behavior. Third, our findings explain the inconsistent and mixed results of previous studies and highlight the findings addressed by the authors of the literature above (e.g., [4, 8, 43, 44]). Finally, most prior studies in developed countries have focused on the relationship between certain board characteristics and IE; for example, Ullah, Zeb [45] and Mirza, Majeed [46] investigated the impact of board diversity on IE; Nor, Nawawi [47] and Salin, Nor [48] examined the impact of board size, board independence, and managerial ownership on IE. Very few studies are available in the local context on board characteristics-IE [49, 50]. In addition to these few studies, no research has been conducted to investigate the moderating effect of IO on the relationships between board characteristics and IE. Our study extends and supplements previous research by focusing on four BoD characteristics in a developing country. The present study indicates to regulators, investors, and shareholders that an effective board of director’s mechanism is fundamental to making a better investment decision.

The current study is structured as follows: section 2 presents the development of corporate governance in Pakistan, literature review and hypothesis development discussed in chapter 3. Chapter 4 covers the research methodology following the result discussion presented in chapter 5. The conclusion is covered in section 6.

## 2. Corporate governance in Pakistan

Pakistan hasn’t been aware of CG for very long [51]. The Securities and Exchange Commission of Pakistan (SECP) is responsible for enforcing corporate governance standards in the country. In March 2002, the SECP issued corporate governance standards in collaboration with the Institute of Chartered Accountants of Pakistan to promote corporate responsibility, openness, and the protection of minority shareholders. In 2012, the SECP updated these mandatory codes to improve openness, transparency, and accountability for businesses [52].

The SECP made a number of changes to previously published codes in 2017 with the publication of the CG codes 2017. According to the updated regulations, a single individual is now permitted to serve as a director for a maximum of five publicly traded companies. At a minimum, a board must contain at least two independent directors, or at least one-third of the board members must be independent; whichever number is greater. The requirement that each listing company must have at least one female director on its board is one of the new revisions to the codes that are intended to encourage the participation of women on corporate boards. In a similar vein, the number of executive directors in relation to total membership shouldn’t be any higher than one-third. Finally, the position of chief executive officer (CEO) and chairman of the board cannot be held by the same individual. In addition, the codes place an emphasis on director training to acquaint them with relevant rules and regulations, applicable laws, as well as their duties and responsibilities, and it is required that every director attend the training program until June 30, 2021.

On September 25, 2019, the SECP released revised codes titled "2019 code." The maximum and minimum limits for independent directors, executive directors, and chief executive officers remaining unchanged in revised codes’ mandatory provisions. The Code of 2019 does not mandate that the board of directors establish a formal mechanism for selecting, monitoring, and overseeing succession planning and executive compensation. In Code 2017 it is emphasized that the board of directors must approve the directors’ compensation policy, but this requirement has been eliminated in more recent codes.

The level of investment efficiency is significantly affected by corporate governance. An efficient and effective governance mechanism serves as an effective check on the organization’s management, thereby significantly enhancing the quality of the organization’s investment decisions. With the publication of revised codes, the quality of government in Pakistan is gradually improving. Therefore, it is reasonable to assume that this gradual improvement in governance quality contributes to the increased investment efficiency of PSX-listed companies.

CG has piqued the interest of Pakistani researchers in recent years. Many researchers have conducted studies on CG, but there is still a need to investigate the relationship between CG and investment efficiency in firm characteristics. In this regard, Mirza, Majeed [46]; Azhar, Abbas [49]; and Shahzad, Rehman [53] have done important work in Pakistan on the relationship between CG and investment efficiency. These studies simply investigate the impact of board characteristics on investment efficiency. While, as previously stated, SECP first issued governance codes in 2002, they were later revised in 2012, 2017, and 2019, with the goal of strengthening the governance structure in PSX-listed firms. As a result, it is critical to assess whether this objective has been met by investigating the relationship between board governance and investment efficiency in the context of different eras of governance codes. This is the goal of the current study. The current study examines the board characteristics-investment efficiency relationship first and then expands the investigation by looking at this relationship in two different eras of corporate governance codes. Finally, in this study, we look at the moderating effect of institutional ownership, which has yet to be tested in the context of Pakistan.

## 3. Review of literature and development of the hypothesis

### 3.1 Board characteristics and IE

According to upper echelons theory, a firm’s behavior reflects its top executives. The board of directors significantly impacts the business’s success and corporate decisions [22]. According to Gul, Srinidhi [54] and Adams and Ferreira [55], effective board monitoring increases corporate efficiency. On the other hand, Ehikioya [56] discovers no correlation between board composition and business performance. Only a few research on the relationship between board composition and IE have been reported in the literature, particularly in emerging markets. However, the few studies that have been conducted have yielded inconsistent outcomes.

#### 3.1.1 Board size

An optimal board size that matches the firm’s characteristics will enhance company performance. Ali [57] states that board size positively correlates with firm size. A larger board would bring together more skills, knowledge, and experiences [58]. According to Abidin, Kamal [59], a larger board size may improve a firm’s performance. This is so that larger boards can devote more time and energy to overseeing management. Nor, Nawawi [47] suggest that in the context of investment decisions, a larger board has an inverse relationship with an investment decision because it has a greater inclination to underinvest. On the other hand, Gill, Sharma [18] conducted research in the Indian manufacturing business and concluded that a larger board is positively connected with an investment decision. Similarly, Nguyen and Dong [60] discovered in a study done in Vietnam that board size is positively associated with a firm’s investment choice. Bzeouich, Lakhal [61] too found a positive impact of board size on IE. Azhar, Abbas [49] examined CG-IE behavior in PSX-listed firms between 2010 and 2015 and discovered, based on GMM results, that board size has no significant effect on IE. According to the most recent governance codes issued on September 25, 2019 (CG codes-2019), there is no requirement for PSX-listed firms to have a certain number of directors on their boards. Based on the existing literature, we formulate the hypothesis as follows:

*H1*: *There is a positive impact of board size on the level of investment efficiency in PSX-listed firms*.

#### 3.1.2 Board independence

An independent non-executive director is a person who has no contractual relationship or family affiliation directly or indirectly in an organization. Kim, Burns [21] claim that independent directors comprise professional consultants to make better corporate decisions and thus increase firm performance. Independent directors encourage more effective governance practices in firms [62]; hence independent directors are more equipped to confront management objectively [63]. Independent directors improve the board’s ability to supervise and give advice by keeping an eye on how management is doing, preventing conflicts of interest, and increasing the BoD’s credibility as a place to make decisions [64]. According to prior research, effective oversight by outsider board members prevents insiders from maximising their benefits and amassing excessive perks, as well as advising them to invest in profitable projects and improve financial report transparency [65]. It improves corporate investment effectiveness. Setia-Atmaja, Tanewski [66] state that independent board members can effectively serve shareholders and protect their wealth, and that agency theory strongly supports this idea. Independent directors make rational decisions and eliminate the possibility of irrational investment decisions from management, increasing the organization’s efficiency and operating performance. Niu [67] argues that independent non-executive directors impact the monitoring and integrity of the financial accounting of an organization. Further, existing studies show that most independent directors on the board negatively influence earnings management [63], minimize accounting fraud cases [68], and save firms from misusing firm resources management. Henry [69] asserted that an independent board helps minimize agency costs and increase firm performance. Chau and Gray [70] and Bzeouic, Lakhal [61] found a direct relationship between board independence and IE, while Nor, Nawawi [47] and Tran [71] fail to find any statistical association between board independence and IE. Based on the literature, we formulate the hypothesis as follows:

*H2*: *There is a positive impact of board independence on the level of investment efficiency in PSX-listed firms*.

#### 3.1.3 Board meetings

It has been argued that more frequent board of directors’ meetings lead to better monitoring and control by the board, which in turn leads to greater financial performance. Vafeas [72] examined the relationship between firm value and board meeting frequency for the first time for 307 companies between 1990 and 1994. He discovered that board meeting frequency is negatively correlated with firm value. According to Zabri, Ahmad [73], the most important CG structure is the board of directors. Regular board meetings have a greater impact on the efficiency and effectiveness of this governance mechanism. Ntim and Osei [74] explain the importance of board meetings by arguing that regular board meetings enhance the advising capacity of the board and bring more control and discipline to the organization, which indirectly increases firm performance. Karamanou and Vafeas [75] found that a board meeting positively correlates with firm performance among 275 publicly traded companies in the United States. Contrarily to the above arguments, literature also witnesses other arguments presented by researchers that regular board meetings result in higher costs, eventually leading to the business’s poor financial position. Similarly, Vafeas [72] proposed an adverse link between board meeting frequency and business performance. Ponnu and Karthigeyan [76], on the other hand, found no significant correlations between them. The following hypothesis will be tested:

*H3*: *Board meetings is positively associated with the level of investment efficiency of PSX-listed firms*.

#### 3.1.4 Board gender diversity

A gender-diverse board brings more expertise and monitoring capacity, enhancing firm performance. Supporting the above argument, Mallin and Michelon [77] added that a gender-diverse board improves board governance by considering diverse stakeholders’ interests and increasing the board’s monitoring function. Ullah, Zeb [45] advocate women’s participation on the board by arguing that it increases the CG mechanism, leading to higher firm performance. Similarly, Arayssi, Dah [78] claimed that greater participation of women on the board strengthens CG mechanisms and raises firm performance. In the same way, Post, Rahman [79] argue that women’s participation on the board brings different knowledge, ideas, and perspectives, which eventually enhance the decision-making process and increase firm performance. In a meta-analysis of 150 studies on "gender differences in risk taking," Hoang, Nguyen [80] found that men take more risks than women. Women invest less and are more risk-averse than men [81]. Levi, Li [82] found that female firm leaders are less aggressive during acquisitions than male leaders. Thus, we expect a gender diverse board to struggle to agree on an investment policy that doesn’t benefit shareholders. Thus, under- or over-investment will be minimised. According to Barber and Odean [83], a board with a diverse gender composition makes better investment decisions and boosts a company’s bottom line performance because female board members are less likely to take unnecessary risks. As a result, it is assumed that the presence of women on corporate boards improves CG and decision-making quality and thus improves investment decisions.

According to Adams and Ferreira [55] and Liao, Luo [84], women on boards make board monitoring better. In this way, businesses make better investment decisions because they have less information asymmetry because of this relationship. Shin, Chang [85] investigated the impact of board gender diversity on IE in a sample of Korean companies. This research spans the years 2006 to 2014. According to the regression results, a more gender-diverse board positively impacts IE. Bzeouich, Lakhal [61] and Ullah, Zeb [45] found that more women on the board made the investment process more efficient. However, Nguyen and Dong [60] fails to find any association between board diversity and company investment decisions. The following hypothesis will be tested from a review of the literature:

*H4*: *There is a positive impact of board gender diversity on the level of investment efficiency in PSX-listed firms*.

### 3.2 Board characteristics and investment efficiency: the role of institutional ownership

Many academics believe that institutional owners have a substantial influence on organizational decisions. Institutional owners have significant voting power and an information advantage over minority shareholders [86]; thus more actively involved in the firm’s decision-making process than non-institutional shareholdings [87, 88]. Furthermore, because institutional investors own a large proportion of the company’s stock, they actively perform their monitoring role [43, 89], and are more interested in the firm’s strategic decisions [90]. Institutional investors have been identified as a key determinant of board characteristics in the empirical literature [91]. According to Mallin [92], if a company’s board of directors is ineffective, IO can either directly express their dissatisfaction with management (the voice option) or sell their stock [93]. On the other hand, institutional investors do not use an exit strategy when they have a large investment and instead try to influence management [94]. Institutional investors can exert influence on management in a variety of ways. Financial institutions, for example, have a direct access with the management of the company in which they have invested [95]. Second, different financial institutions within a firm may band together to form a representative group, which can interact with management on behalf of the financial institutions [96]. Third, if the governing body fails to perform its duties and violates CG principles, it may file a lawsuit against it [97]. Fourth, unlike individual investors, institutional investors exercise their voting power wisely based on their knowledge, skills, and ability [98]. As a result of voting rights, financial institutions gain explicit and implicit powers, which they use to select or dismiss board members at the Annual Shareholder’s Meeting [99].

Furthermore, institutional investors are pressuring management to change executive compensation to align shareholders’ and management’s interests [100]. Board size is a significant deterrent to IE and an important component of institutional investment [101]. Institutional investors prefer firms with a smaller board size and a higher ratio of independent directors, according to Bushee, Carter [102]. Similarly, Nwaiwu [103] found that board size and institutional investment have an inverse relationship in developing countries.

Institutional investors strengthen the governance mechanism by increasing board independence and separating the chairman and CEO positions [104]. Similarly, according to Schnatterly and Johnson [105], institutional investors prefer to invest in companies with a majority of independent directors and no duality between the chairman and CEO. IO is related to board independence, while managerial ownership is inversely related. Because of poor governance, institutional investors are less likely to participate in a company’s ownership structure [30]. Thus, the following hypothesis can be developed based on the arguments:

*H5*: *Institutional ownership moderates the relationship between board characteristics (board size*, *board independence*, *board meetings*, *and board gender diversity) and the level of investment efficiency in PSX listed firms*.

### 3.3 Theoretical framework

Based on the foregoing discussion, Fig 1 below depicts the conceptual framework of the current study.

**Fig 1:** Conceptual framework.

## 4. Research methodology

### 4.1 Population and sample

The preliminary sample for this study consists of all firms listed on the Pakistan Stock Exchange (PSX) as of June 30, 2018, i.e. 544. The sample of the research spans the years 2004 to 2018. 2004 has been designated as the base year. The rationale is that Pakistan issued its first governance codes in March 2002. It is anticipated that the same will be incorporated into their annual reports for 2004. Financial firms were excluded from the data set due to their differences in regulatory requirements and business nature [106]. Consequently, 135 financial firms were eliminated from the initial sample, leaving 409 remaining. In addition, thirteen state-owned companies were eliminated, reducing the sample size to 396. To become a part of the study, firms must meet the following criteria:

- Firms remain listed during the whole study period.
- All required variables data should be made available.
- There is not any merger or acquisition of the firm during the study period.

Companies that consistently lost money throughout the duration of the study were eliminated from the study. As a result, further 241 non-financial firms were eliminated from the sample using these filtering techniques, leaving 155 non-financial firms. Hence the final sample of the study comprises of 155 non-financial firms (2,325 firm-year observations). The distribution of the sample across the industry is presented in Table 1. To obtain the desired variable data, various sources were used. The annual reports of respective companies are a major source of data collection. Additional data were gathered from SBP financial statement analysis, the SECP official data site, and brecorder.com. Industry-wise sample detail is presented in Table 1.

**Table 1:** Industry-wise sample distribution.

Industrial Sectors	No. of Firms	% of Sample
Automobile and Parts	16	10.19
Cable & Electrical goods	3	1.91
Cement	10	6.37
Chemicals	15	9.68
Engineering	2	1.27
Fertilizers	1	0.64
Food & Personal care	15	9.55
Glass & Ceramics	5	3.18
Leather	2	1.27
Miscellaneous	4	2.55
Oil & Gas	14	8.92
Paper & Board	4	2.55
Pharma	5	3.18
Power	5	3.18
Sugar	20	12.74
synthetic & Rayon	4	2.55
Telecom	5	3.18
Textile Comp	23	14.65
Transport	2	1.27
**Total**	**155**	**100**

According to the table, the textile sector has the highest representation in the sample firms, at 14.65 percent, followed by the sugar and chemical sectors, at 12.74 percent and 9.68 percent, respectively. The transportation and engineering sectors have the lowest representation in sample firms, accounting for 1.27 percent each. Following Farooq and Noor [107], we winsorized all continuous variables @ 1% and 99% to remove the effect of the outliers.

### 4.2 Measurement of variables

#### 4.2.1 IE

To test the hypotheses, we follow Biddle, Hilary [8] and estimate the level of investment in the upcoming year as a function of growth opportunities in the current year. The investment model is described below:

$$Investment_{i,}=\beta 0+\beta 1Sales\;growth_{i,―1}+\varepsilon_{it}$$ (1)

Where is the aggregate investment_*it*_ investment of firm *i* in year *t*, measured as the net increase in tangible and intangible assets and deflated by lagged total assets? Sales growth_*i*,― 1_, a proxy for investment opportunities, is the annual sales growth firm *i* from t—2 to year *t*.

Board governance mechanisms of sample firms can be measured using board size, board independence, board meetings, and board gender diversity. Further, firm size, leverage, and ROA are used as control variables. Table 2 explains the symbol and measurement of variables.

**Table 2:** Description of variables and data sources.

Name	Symbol	Description	Source
**Independent Variables**			
Board Size	Bsize	Measures by total number of directors in board	Annual Report
Board Independence	Bind	Measures by proportion of independent directors to total number of directors in board	Annual Report
Board Activity	Bact	Number of board meetings in a financial year	Annual Report
Board Diversity	Diversity	Measures by 1 in case of presence of woman director in board; 0 otherwise.	Annual Report
Institutional ownership	Inst_Own	Fraction of shares held by institutions	Balance Sheet Analysis
**Control Variables**			
Firm Size	Fsize	Log of total assets	Balance Sheet Analysis
Leverage	Lev	Total debt/Total assets	Balance Sheet Analysis
Firm’s profitability	ROA	Net income/Total assets	Balance Sheet Analysis

#### 4.2.2 Board characteristics

The main explanatory variable in the study is board characteristics. We measured the board governance structure using four board governance characteristics, namely board size, board independence, board meetings, and board gender diversity, which are consistent with the existing literature (e.g., [4, 19, 22, 107, 108]). The current study assesses the board governance mechanism of sample firms using four proxies: board size, board independence, frequency of board meetings per year, and board gender diversity. Table 2 contains information about how to measure these variables.

#### 4.2.3 Control variables

Several other variables are used as control variables, which may influence investment decisions. The first control variable is firm size, which is calculated by taking the log of total assets. According to Himmelberg, Hubbard [109], firm size is an efficient monitoring mechanism that limits management’s opportunistic behavior because larger firms have better technology, greater diversification, and competent management. According to Kadapakkam, Kumar [110], firm size can influence a firm’s investment decision. As a result, we can control firm size. Furthermore, we account for leverage, as agency theory explains that leverage is a monitoring mechanism that limits management’s opportunistic behavior [9]. Aivazian, Ge [111] also argued that leverage has a negative impact on investment efficiency and that we should account for it. Our third control variable is profitability. Ullah, Zeb [45] used return on assets (ROA) as a control variable in their respective studies, claiming that it can potentially influence investment decisions. Furthermore, Chen, Sung [4] investigated the relationship between corporate governance and investment efficiency in Chinese firms, using firm size, leverage, and profitability as control variables to account for the effect of financial status on investment efficiency. In empirical studies of corporate finance, including control variables in regression has been a preferred method of avoiding potential endogeneity problems [22].

### 4.3 Econometric model

The panel data model was used. It’s best employed in social science research since it produces more reliable results than other methods [112]. Individual variability is captured by cross-sectional data, whereas time-series data show variations within subjects across time [113]. The model is expressed as follows:

$$IE_{it}=\alpha_{0}+\beta_{1}Bsize_{it}+\beta_{2}Bind_{it}+\beta_{3}Bact_{it}+\beta_{4}Diversity_{it}+\beta_{5}Fsize_{it}+\beta_{6}ROA_{it}+\beta_{7}Lev_{it}+\varepsilon_{it}$$ (2)

The moderating impact of IO can be tested through the following model:

$$IE_{it}=\alpha_{0}+\beta_{1}Bsize_{it}+\beta_{2}Bind_{it}+\beta_{3}Bact_{it}+\beta_{4}Diversity_{it}+\beta_{5}Inst\_own_{it}+\beta_{6}Bsize_{it}*Inst\_own_{it}+\beta_{7}Bind_{it}*Inst\_own_{it}+\beta_{8}Bact_{it}*Inst\_own_{it}+\beta_{9}Diversity_{it}*Inst\_own_{it}+\beta_{10}Fsize_{it}+\beta_{11}ROA_{it}+\beta_{12}Lev_{it}+\varepsilon_{it}$$ (3)

### 4.4 Econometric methodology

The data set was first subjected to pooled regression to determine whether all of the firms under consideration were the same. A Durbin-Watson score of 0.20 indicates that the model is susceptible to autocorrelation. It means that the model did not adequately fit the data [113]. The problem was solved using a more complex regression method panel estimation technique. The Hausman test was used to determine which regression model best suited the data. The Hausman probability value prefers the random effect model. Furthermore, corporate governance (board governance) is endogenous, which means that firms with different types of directors on their boards exhibit different characteristics. Fixed-effects models are frequently inconclusive. As a result, we used the random-effect model to summarize the findings of the study.

## 5. Empirical results

### 5.1 Descriptive results

Descriptive statistics are presented in Table 3. The mean value of IE is -0.088, with a standard deviation of 0.072. The sample firms have an average of 8 members on their boards, with a range of 7 and 12 members, respectively. 40% of the board members are independent directors, with a 5% minimum and 91% maximum independent directors, respectively. Five board meetings were held in sample firms during a fiscal year. Female directors make up 28% of the board. Institutional owners own 11% of the sample firms on average. IO’s minimum and maximum levels are 0 percent and 35%, respectively. The average ROA for sample firms is 11.5 percent, with minimum and maximum profit earnings of -0.048 and 0.33, respectively. The average leverage value is 0.538, with a standard deviation of 0.206. This highest mean value of leverage indicates that Pakistani firms are leveraged, which raises the risk of financial distress. Table 4 shows the correlations between variables. The results show that there is no problem with multicollinearity among firms because no value exceeds the threshold level of multicollinearity. As a result, our data is free of multicollinearity among variables.

**Table 3:** Descriptive statistics.

Variable	Obs	Mean	Std. Dev.	Min	Max
**IE**	2354	-.088	.072	-.323	-.01
**Bsize**	2355	8.193	1.512	7	12
**Bind**	2355	.408	.293	.057	.909
**Bact**	2355	5.236	1.42	4	9
**Diversity**	2355	.288	.457	0	2
**Inst_own**	2355	.116	.106	0	.351
**Fsize**	2348	9.698	.669	8.495	10.934
**ROA**	2348	.115	.099	-.048	.33
**Lev**	2352	.539	.206	.173	.898

**Table 4:** Matrix of correlations.

Variables	(1)	(2)	(3)	(4)	(5)	(6)	(7)	(8)
Bsize	1.000							
Bind	0.193	1.000						
Bact	0.146	0.143	1.000					
Diversity	-0.071	-0.144	0.051	1.000				
Inst_os	0.101	0.141	-0.028	-0.144	1.000			
Fsize	0.344	0.227	0.254	-0.109	0.062	1.000		
ROA	0.118	0.029	-0.020	-0.067	-0.013	0.151	1.000	
Lev	-0.016	-0.015	0.028	0.037	-0.032	-0.003	-0.373	1.000

### 5.2 Regression results

As previously discussed, we used the Hausman test to select the best model for the analysis. The Hausman test results, presented in Table 5, (p-value>0.05, i.e., 0.7343) favored the REM as the best model to analyze the impact of board characteristics on IE. Table 6 displays the results of the REM. The value of R-square is moderately low in model 1 and 2 i.e. 0.1215 and 0.1391 respectively, but it is common in corporate governance studies. As Rehmat and Iskandar [114] mentioned on page 9 as follows: “*Results show the value of R-square is 0*.*047 for the basic regression of test variables*, *which is moderately low*. *This low in R-square is common in studies examining corporate governance characteristics*”. Board size is the first variable of board characteristics which shows a significant positive association with IE. Results support the findings of Gill, Sharma [18], Nguyen and Dong [60], and Bzeouich, Lakhal [61], who argue that larger board sizes are positively associated with a firm’s investment decisions. Moreover, many studies show board size is positively linked with firm performance, like Dalton, Daily [115] and Kiel and Nicholson [58]. In a local context, Nazir and Afza [19] proposed that board size has a positive impact on firm performance. This positive association supports the findings of Khattak, Hussain [116] who studied the relationship between corporate governance and investment efficiency in 56 non-financial firms and discovered that board size is positively associated with IE. This supports the argument that a larger board provides greater skills, knowledge, and expertise and puts effective monitoring on management, increasing firm IE in PSX listed firms.

**Table 5:** Hausman test results.

	Full Sample	Before 2012	After 2012
Chi2(10)	6.91	10.88	5.21
Prob>chi2	0.7343	0.2840	0.8160
Decision	Random Effect Model	Random Effect Model	Random Effect Model

**Table 6:** Regression results.

Variables	Model 1	Model 2	Robustness test
	REM	REM	REM
**Bsize**	0.00297**	0.00258*	0.00211**
	(0.001)	(0.002)	(0.002)
**Bind**	-0.00313	-0.0199	-0.00942
	(0.006)	(0.009)	(0.007)
**Bact**	-0.00285**	-0.00400**	-0.00335**
	(0.001)	(0.002)	(0.001)
**Diversity**	0.00148	0.000305	0.00176
	(0.004)	(0.005)	(0.005)
**Inst_own**		0.129**	
		(0.099)	
**Bsize** * **Inst_own**		0.00082*	
		(0.011)	
**Bind** * **Inst_own**		0.132**	
		(0.054)	
**Bact** * **Inst_own**		0.0104*	
		(0.011)	
Diversity*Inst_own		0.00683	
		(0.037)	
**Fsize**	0.00866***	0.00846***	0.00852*
	(0.003)	(0.003)	(0.005)
**ROA**	0.0753***	0.0734***	0.0588***
	(0.019)	(0.019)	(0.021)
**Lev**	-0.00653	-0.00749	-0.00179
	(0.009)	(0.009)	(0.011)
**Constant**	-0.186***	-0.166***	-0.226***
	(0.030)	(0.032)	(0.045)
**Observations**	2,347	2,347	2347
**No. of Firms**	157	157	157
**R-square**	0.1215	0.1391	0.106
**Wald-chi(12)**	44.68	53.3	20.81
**Prob>chi2**	0.0000	0.0000	0.0041

Note: Standard errors in parentheses

*** p<0.01

** p<0.05

* p<0.1

Board independence shows an insignificant association with IE. This insignificant association witnessed that Pakistani firms lack board independence in real means. As family businesses are prevalent in Pakistan, family members nominate friends or family members as independent directors; hence they are not truly independent. Resultantly they cannot participate more actively in business decisions like investment decisions of an organization. This shows an insignificant association with an investment decision. This insignificant relationship supports the findings of Nor, Nawawi [47], Chen, Sung [4], and Salin, Nor [48]. Khattak, Hussain [116] fail to find any significant impact of board independence on IE in a local context.

Board activity presents a significant negative association with IE among sample firms. This shows that the meeting frequency in a local context is not as effective as it should have been. This supports the argument of Yasser [117] and Nazir and Afza [19], who suggested that meeting frequency has a significant inverse relationship with firm profitability. The cost of holding board meetings, including director fees, travel expenditures, refreshments, and managerial time, could be the reason for this negative association, resulting in decreasing value [72]. This significant negative relationship demonstrates that directors hold meetings solely to comply with regulations or for the sake of formality. They are not well prepared, and agenda items are not shared ahead of time, so this activity has no impact on investment quality decisions. Among other board characteristics, diversity fails to impact IE in Pakistani firms. Results align with Mirza, Majeed [46], who found that diversity is insignificantly associated with IE in Pakistani firms. This insignificant association suggests that either women board members face barriers to actively participating in board activities or do not currently have the necessary skills and expertise to play an active role on the board.

Regarding control variables, firm size and ROA were discovered to be positively related to IE. The larger the firm and the greater its profitability, the better the firm’s investment decision. Nor, Nawawi [47] discovered a link between firm size and investment behavior. Leverage was found to be insignificantly related to IE. This backs up the findings of Mirza, Majeed [46] and Agyei-Mensah [22].

After investigating the impact of board characteristics on the IE of PSX-listed firms, we extend our analysis to investigate the moderating impact of IO in this relationship. Table 5 shows the results. The findings show that IO significantly moderates the relationship between board size and IE. Furthermore, IO significantly moderates the relationship between board independence and IE in a positive way. Earlier results show that board independence does not affect IE. This significant positive moderating impact demonstrates that having an institutional owner representative on the board as an independent director improves board efficiency. As a result, board independence increases the firm’s IE. This supports the argument that institutional owners have greater expertise, experience, and financial stake in the investee firm, so they actively monitor management, resulting in improved board performance. In line with the preceding argument, IO significantly moderates the relationship between board activity and IE. The number of board meetings increases the board’s efficiency when there is an IO representative. As a result, it significantly impacts the quality of the firm’s investment decision. Finally, IO has no significant impact on the relationship between board diversity and IE.

### 5.3 Robustness test

To assess the robustness of the findings, the dependent variables, namely IE, are calculated by including profitability as a growth opportunity factor in Eq 1. Bimo, Silalahi [118] use the same proxy to test the effect of CG on IE empirically. As a result, the following equation model is used to calculate the IE.

$$InvEff_{it}=\beta_{0}+\beta_{1}SalesGrowth_{i,t‐1}+\beta_{2}ROA_{i,t‐1+}\varepsilon_{it‐1}$$ (4)

The test results, as shown in Table 6, support our main regression analysis findings. The results back up the fact that board size has a significant positive relationship with IE, while board meetings have a significant negative relationship with IE. The remaining board characteristics, namely board independence and board diversity, do not affect the IE of the sample firms.

Endogeneity problems in regression models can also be caused by omitted variable bias (including variables like board room experience, skill, and education), measurement error, and simultaneous/reverse causation. Endogeneity would make the OLS, fixed effect, and random effect not match up, which would lead to an unfair result. Because we didn’t have a valid instrument, which is a requirement of the 2SLS, we used the Generalized Method of Moments (GMM) to estimate. Dynamic GMM models come in two forms: differenced GMM and system GMM. When the sample size is big, you should use a two-step difference GMM [119]. So, we used a different GMM with a two-step process.

The models are defined then following ways:

$$IE_{it}=\alpha_{0}+\beta_{1}Bsize_{it}(‐1)+\beta_{2}Bind_{it}(‐1)+\beta_{3}Bact_{it}(‐1)+\beta_{4}Diversity_{it}(‐1)+\beta_{5}Fsize_{it}(‐1)+\beta_{6}ROA_{it}(‐1)+\beta_{7}Lev_{it}(‐1)+\varepsilon_{it}$$ (5)

In two-step difference GMM, we used the first difference of all independent variables as an independent variable, along with the lagged dependent variable. The Wald test is a Chi-square distribution that measures how important the independent factors are in relation to the dependent variable as a whole. In the first-difference residuals, AR(1) and AR(2) are used to check for the lack of first-order and second-order serial correlations, respectively. J-statistics is a type of the Sargan test that is used to find out if an instrument is reliable. The results shown in Table 7 support our main findings which are presented in Table 6.

**Table 7:** GMM Regression results.

IE	Coef.	St.Err.	t-value	p-value	[95% Conf		Interval]	Sig
Log (IE)	.078	.02	3.84	0	.038		.117	***
Bsize (-1)	.002	.003	0.46	.064	-.005		.008	*
Bind(-1)	.019	.012	1.55	.121	-.005		.043	
Bact(-1)	-.004	.002	-1.88	.06	-.008		0	*
Diversity(-1)	-.007	.008	-0.85	.396	-.022		.009	
Inst_own(-1)	.088	.04	2.19	.029	-.166		.009	**
Fsize(-1)	.015	.011	1.41	.159	-.006		.036	
ROA(-1)	.029	.034	0.83	.404	-.039		.096	
Lev(-1)	.01	.021	0.46	.649	-.032		.051	
Constant	-.07	.032	-2.23	.026	-.132		-.008	**
Mean dependent var	-0.088		SD dependent var			0.071		
Number of obs	2196		Chi-square			30.592		
AR(1)	0.0000		J-statistics			53.38		
AR(2)	0.445							

*** p < .01

** p < .05

* p < .1

### 5.3 Additional analysis

After investigating the impact of board characteristics on the IE of PSX sample firms, we broaden our analysis by dividing the sample into two periods, 2004 to 2013 and 2014 to 2018. This division of the sample is since SECP issued the code of CG first time with the collaboration of ICAP (Institute of Chartered Accountants of Pakistan) on March 28, 2002, and later on, SECP revised these codes to further strengthen the governance structure in the PSX listed firms on April 2012. It would be interesting to investigate the relationship between board characteristics and IE in these two periods to understand better how board mechanisms impact IE in the initial phase (2004–2013) and later in the revised phase of CG (2014–2018).

Awareness of CG is a relatively new phenomenon in Pakistan. SECP issued CG codes first time in March 2002, which was mandatory for publicly listed firms in Pakistan. This code establishes "best corporate practices" following the provisions of the Companies Ordinance 1984. SECP modified the CG code in revised CG codes (2012) to strengthen the CG board mechanism further. Several initiatives have been undertaken; for example, in revised codes, one board member must be an independent director, whereas, in the introductory phase, this is not required.

Similarly, in revised codes, executive directors should not constitute more than one-third of the board of directors, while previously, executive directors should not constitute more than seventy-five percent. Similarly, in revised codes, the CEO and chairperson cannot be the same person, whereas, in the initial phase, the same person may hold both positions. The revised codes give the board the authority to choose the chief financial officer and company officer, whereas the previous CEO could choose the chief financial officer and company secretary. Table 8 contains a summary of governance code changes between 2002 and 2012. As a result, it is critical to investigate the impact of these governance improvements on the IE of PSX-listed companies.

**Table 8:** Comparison of 2002 and 2012 codes.

S. No	Issue	Code 2002	Code 2012
1	Independent director	Encourage minimum one independent director in board	One is mandatory while preference is 1/3 of members to be independent.
2	Executive director	Not more than 75% of the board including CEO	Cannot be more than 1/3 of elected director including CEO
3	No. of directorship	Not more than 10 listed Companies at any time.	Not more than 7 listed companies in any time.
4	Board evaluation	-	Within two years of the implementation of code 2012, board define mechanism to check performance of the board
5	Office of the chairman and CEO	Chairman preferably elected among non-executive directors of listed company	CEO and Chairman shall not be the same person.
6	Training of the board of directors	Mandatory for directors	Mandatory.
7	Appointment and removal and qualification of CFO and CS	Determined by the CEO and approved by the board	Determined by the board CFO stand for chief financial officer CS stand for company secretary
8	Head of Internal audit	-	Qualification introduced. Removal with the approval of the board only on the recommendation of chairman of audit committee.
9	Remuneration of directors	-	Mentioned in annual report
10	Board committees	Audit committee: chairman preferable non-executive director	Audit committee: chairman shall be independent director. Comprises non-executive directors.
11	Internal audit	Shall be internal audit in every listed Co. Head of internal audit shall have an access to chairman of audit committee.	Internal audit function may be outsourced by a listed company to a professional services firm or staff of holding CO.

We begin our analysis by comparing the descriptive statistics of the variables studied between these two governance phases. Table 9 shows the results. According to the findings, the level of IE has increased since the issuance of CG codes in 2012, and in the same way, the level of board independence and diversity has also increased from 0.384 to 0.443 and from 0.273 to 0.318, respectively. Further, a paired sample t-test was performed on IE before and after the CG codes 2012 to determine whether there was a significant improvement in IE. The results show a significant increase in IE from -0.095 to -0.079 after the issuance of revised codes. (See Table 10). The average IE is -0.088, with values ranging from -0.322 to -0.010. These findings support previous research by Chen, Hope [17] and Gomariz and Ballesta [37].

**Table 9:** Descriptive statistics (2004–2013) & (2014–2018).

Variables	(2004–2013)			(2014–2018)		
	Obs	Mean	Std. Dev.	Obs	Mean	Std. Dev.
**IE**	1569	-0.093	0.079	785	-0.078	0.055
**Bsize**	1569	8.159	1.489	785	8.262	1.553
**Bind**	1569	0.384	0.298	785	0.455	0.275
**Bact**	1569	5.227	1.414	785	5.253	5.253
**Diversity**	1569	0.273	0.445	785	0.318	0.318
**Fsize**	1569	9.598	0.655	778	9.899	0.652
**ROA**	1569	0.121	0.098	778	0.105	0.1
**Lev**	1569	0.548	0.201	782	0.519	0.212

**Table 10:** Paired-samples t-test for pre and post CG code 2012.

Mean Investment efficiency Post CG-code 2012	Mean Investment efficiency before CG-code 2012	Paired differences				
		Mean	SD	SE mean	t-statistics	Significance
-0.079	-0.094	0.015	0.073	0.003	5.052	0.000

Finally, we conducted a regression analysis to determine the impact of board characteristics on IE during these two distinct phases, i.e., 2004 to 2013 and 2014 to 2018. To select the most suitable model for the analysis, we applied the Hausman test (results are presented in Table 11). Based on the Hausman test, we used REM to conclude. Results are presented in Table 12. Result shows that there are no significant differences in the impact of board characteristics on IE across both sample periods, except board diversity, which significantly positively impacts IE from 2014 to 2018. Because board diversity increased following the adoption of revised codes, as previously discussed, this strengthened board governance and positively impacted IE. Although there has been an increase in the level of board independence, it has failed to demonstrate any positive impact on IE. This demonstrates that, while there are independent directors on the board to comply with the CG codes-2012, they are not truly independent. There is a need to further strengthen the governance mechanism in PSX-listed firms to reap the benefits of higher investment efficiency and profitability.

**Table 11:** Hausman test results.

	2004–2013	2014–2018
**Chi2 (11)**	10.73	6.76
**Prob>chi2**	0.4664	0.8185

**Table 12:** Regression results.

Investment Efficiency	(2004–2013)	(2014–2018)
	REM	REM
**Bsize**	0.00394**	0.00341**
	(0.002)	(0.002)
**Bind**	-0.00706	-0.00925
	(0.008)	(0.008)
**Bact**	-0.00228*	-0.000439*
	(0.002)	(0.002)
**Diversity**	-0.00523	0.00789*
	(0.005)	(0.005)
**Fsize**	-0.00175	0.0101**
	(0.004)	(0.004)
**ROA**	0.104***	0.0342
	(0.025)	(0.025)
**Lev**	0.00524	-0.0175
	(0.012)	(0.012)
**Constant**	-0.131***	-0.201***
	(0.043)	(0.042)
**Observations**	1,569	778
**Number of coid**	157	157
**R-Sq**	0.1529	0.165
**Wald-Chi2**	36.91	33.32
**Prob>Chi2**	0.0001	0.0005

Note: Standard errors in parentheses

*** p<0.01

** p<0.05

* p<0.1

## 6. Conclusions

The current study aims to examine board characteristics’ impact on IE of 155 PSX-listed firms from 2004 to 2018. The role of IO has also been investigated in the context of the board characteristics-IE relationship. Another significant contribution of this study is that we divide the sample into two groups, the introductory phase of CG (2004 to 2013) and revised codes of CG-2012 (2014–2018), to study the level of IE of sample firms separately. Furthermore, we investigate the board characteristics-IE relationship in both periods to understand better the role of revised codes in strengthening the board governance mechanism among sample firms. Following Biddle, Hilary [8], we measure IE regarding growth opportunities. Board governance mechanisms are measured by board size, independence, activity, and diversity, with firm size, leverage, and ROA used as control variables. Based on the Hausman test result, REM is used to conclude the study’s findings. First, the effect of board characteristics on IE is investigated. Regression analysis showed that board size positively affects IE, while board activity negatively affects it. Board independence and board genders diversity fails to show any significant impact on IE. The influence of IO on the effectiveness of IE is significant and positive. Additionally, it was found that IO plays a significant role in moderating the positive relationship that exists between board independence and IE. This demonstrates that IO increased the level of independence of the board of directors, which positively impacted IE.

To broaden our analysis, we look at the level of IE of sample firms from 2004 to 2013 and 2014 to 2018. According to t-statistics, there is a significant increase in the level of IE in the later period. Furthermore, it was discovered that board independence and diversity increased after the issuance of the revised code in PSX-listed firms. Finally, we conducted a regression analysis to test separately the board characteristics-IE relationship between two sample periods. We discovered that there is no change in the impact of board characteristics on IE except board diversity, which positively impacted IE from 2014 to 2018. There is a need to strengthen governance mechanisms in the true sense so that firms can reap the benefits of increased profitability and IE. The current study’s empirical result adds to the existing literature by investigating the effect of board characteristics on IE in various governance eras.

The study’s findings provide important evidence for investors, top management, planners, and future scholars. The research benefits investors in a variety of ways. The size of the board and the level of IO are both positively related to the level of IE. Before investing in PSX-listed companies, investors must consider these two factors. Furthermore, because board independence is unrelated to IE, investors must scrutinise board independence to ensure that independent directors are truly ’independent.’ The SECP is concerned that board independence has no discernible impact on IE. In Pakistan, the majority of board members lack true "independence." Because the majority of businesses are family-owned. They appoint independent directors to the board in order to meet the governance requirements, but in reality, all board decisions are dominated by the family owners. As a result, it was necessary to issue some guidelines by the SECP for the induction of independent directors to the board in order for independent directors to be truly independent and perform their fiduciary role more independently. Since board diversity has failed to have a significant impact on IE, which is also a major concern for SECP. SECP should develop some policy guidelines regarding the qualifications and experience required for female board members. As a result, the firm truly benefits from board diversity in terms of higher IE. Furthermore, the results show that IO strengthened the board governance mechanism through effective monitoring. As a result, the regulator should take steps to encourage IO to invest in firms. It is recommended that stakeholders consider the board characteristics and level of IO in the respective firm before entering into any relationship with the firm. In the future, the current study could be strengthened by incorporating other CG indicators such as block shareholders, percentages of insider holdings, and the presence and quality of CG committees, as well as investigating their impact on IE. Future research may look into other aspects of financial management decisions. Further evidence from PSX-listed firms suggests a possible bias in the relationship between board qualifications and investment decisions, limiting the findings’ applicability to other countries. Lastly, a cross-country analysis can be conducted from the perspective of board characteristics-IE relationship.
